# Cost Early-Warning Model System of Large-Scale Construction Project

**DOI:** 10.1155/2022/3541803

**Published:** 2022-05-10

**Authors:** Jingyi Dai, Dandan Ke

**Affiliations:** School of Resources and Architectural Engineering, Gannan University of Science and Technology, Ganzhou 341000, Jiangxi, China

## Abstract

China's construction industry has been suffering from high cost, high efficiency, and maladjustment of management. The traditional management mode makes the construction project face the risk of cost overruns and delays, which cannot achieve the effect of cost control. Therefore, by summarizing the characteristics of construction projects and the classification of costs, this paper analyzes the foundation of earned value management method in construction and combines it with cost management; in addition, the actual development of Company A is taken as an example, where a cost early-warning system suitable for construction projects is constructed, including the design of the organizational structure, operation platform, and early-warning model of this system, which can improve the cost management level of construction enterprises to a certain extent.

## 1. Introduction

With China's economy entering a new normal and structural adjustment steadily, the growth target of the total output in the construction industry from 2016 to 2021 is only set at 7%, which reveals that the country's expectation for the construction industry has shifted from the rapid growth in scale in the past to paying attention to the quality of construction projects. In the critical period of transformation and development, the sooner a construction enterprise abandons the growth model driven by low cost in the past and turns to the pursuit of more reasonable internal control process and more accurate cost management process, the more it can seize the opportunity to realize the growth of profit [1].

With the development of new buildings, project management is becoming more and more difficult. For a long time, due to the backward technical means and the lack of modern information management platform in China, the traditional management mode often leads to the risk of cost overruns and schedule delays for most projects, which cannot achieve the effect of cost control [2, 3]. In cost management, the deviation between the budgeted cost and the actual cost is viewed in isolation, the construction progress is not taken into account, the cost management and progress monitoring are not effectively combined, and the management efficiency and cost management effect need to be improved. In addition, the cost management system is imperfect, and most of the cost management systems adopt timing analysis, which cannot realize the timely warning of the cost, which is more of an after-the-fact analysis that makes suggestions on the future cost management, lacking a whole-process dynamic cost early-warning system [4]. The division of responsibility for cost management is unclear, the enthusiasm of all staff for cost management is not mobilized, the participation is low, the coordination among various departments is less, and there is a lack of effective communication. When there are cost management problems, there are many cases where departments shirk their responsibilities. The responsible person cannot be found.

The theory of project cost management can already meet the development needs of daily work, but the research and development of this software still has a lot of room for development due to the complicated projects, huge data processing, multiparty collaboration, and information sharing [5]. Therefore, this paper makes use of the earned value management method to design a system that can realize cost early warning, which combines cost management with progress monitoring and assigns responsibility to people by distributing early-warning instructions, so as to strengthen employees' awareness of cost management, improve the cost management level of enterprises, and increase the company's economic benefits.

## 2. Introduction of Construction Project Cost

### 2.1. Characteristics of Construction Projects

The construction project is a fixed asset investment led by the construction unit and implemented by the construction enterprise. Its process takes effect from the date of bidding and ends with the expiration of the warranty period. Compared with ordinary projects, it also has similar characteristics of definite objectives, irreversible management process, and limited by external environmental conditions. Besides, it has its own uniqueness: (1) large investment in construction projects, (2) long construction plan period, (3) more uncertain factors and risks, (4) large number of participants, etc. [6, 7].

Figure 1 shows the management of the whole construction process including (1) management in the decision-making stage, (2) management in the implementation stage, and (3) management in the use (operation) stage [8, 9]. Among them, the implementation stage of construction projects includes design preparation, design, construction preparation, construction, and acceptance [10].

### 2.2. Composition of Construction Project Cost

There are many classification methods of construction cost, which are generally classified according to different standards and different application scopes. At present, the main classification methods are the cost valuation quota method and the project completion degree method [11].

#### 2.2.1. Classification of Cost Valuation Quota Method

- Budget cost: the average social cost or enterprise cost calculated according to the physical quantity of construction and installation projects and the budget quota and charging standard formulated by the country or region or enterprise are determined by analysis, prediction, collection, and calculation based on the working drawing estimate
- Target cost: according to the requirements of the enterprise itself, such as the provisions of the internal contract, the standard cost, also known as the target cost, is determined by combining the technical characteristics, physical and geographical characteristics, labor quality, and equipment conditions of the construction project
- Actual cost: the sum of all expenses actually incurred during the construction of the project that can be included in the cost expenditure

#### 2.2.2. Classification of Project Completion Degree Method

- Current period construction cost represents all construction costs incurred in the construction of the project during the cost calculation
- Current period completed construction cost represents the partial project cost of which all the contents specified in the budget quota have been completed during the cost calculation period
- Uncompleted construction cost represents the partial project cost of the unfinished budget quota during the cost calculation period
- Completion construction cost represents the cost of the completed unit project during the whole construction period from commencement to completion

## 3. Application Basis of Earned Value Management in Construction

Earned value management is a management method that integrates scope, schedule, and resources to objectively measure project performance [12, 13]. On the basis of work breakdown, a set of methods combining progress monitoring and cost management is established; the project schedule, progress, and cost budget are determined according to the project schedule; and the cost budget is allocated to monitor the progress of the project [14]. Due to the inconsistency between the measurement units of schedule and cost, earned value management method considers converting time scale into monetary scale according to calculation rules and adopting the same index system to measure the performance of project schedule and cost at the same time so as to solve the difficulty that schedule and cost cannot be checked synchronously [15–17]. It is also possible to collect and sort out the data on work progress and cost related to the project at an appropriate time and analyze the next plan of construction implementation and cost management measures according to the results.

### 3.1. Basic Indicators

As shown in Figure 2, earned value management has three basic indicators, namely, BCWS (budgeted cost of work scheduled)[18, 19], BCWP (budgeted cost of work performed) [20–22], and ACWP (actual cost of work performed) [23, 24].

Earned value method will measure and analyze various indicators in cost control so that it can monitor the status of the project in real time, know the relevant cost information at the first time, know the progress trend of the project, and constantly adjust the corresponding measures during the project implementation to ensure that the project cost is within the controllable normal range. The measurement relationship of each index is shown in Table 1.

## 4. Design of Cost Early-Warning System

Company A was founded in 1956, and its construction scope covers many fields such as housing construction, municipal engineering, mechanical, and electrical engineering and participates in the construction of EPC project and PPP project. By taking Company A as an example, in this paper, the cost management of its construction project is analyzed, and a cost early-warning system is built. Through the analysis of the main problems existing in the cost management of the construction project of Company A, some prominent problems are exposed in its cost management: therefore, it is necessary to introduce the cost early-warning system into the cost management.

### 4.1. Organizational Structure Design of Cost Early-Warning System

#### 4.1.1. Establish a Cost Management Center

Company A's cost management system is imperfect, and the division of rights, responsibilities, and benefits is unclear, which leads to the widespread phenomenon that the management departments of Company A pay insufficient attention to cost management. Most departments lack communication, and cost management mainly focuses on the comparison of the difference between budget cost and actual cost, neglecting to find effective strategies, which restricts the development of the construction industry [25–28]. Therefore, it is urgent to strengthen the attention of each management department, establish an effective internal control mechanism of enterprises, and cultivate the consciousness of cost management among all employees. It is suggested that Company A set up a cost management center and choose a new method, which can respectively deploy personnel from the presettlement management center, the engineering management department, the human resources department, the finance department, and the audit department to perform the following main duties:

1. Formulate cost management standards: including compiling the standard manual of cost management, drawing up the detailed implementation rules for full participation, and further improving the construction of the cost management system and internal control system.
2. Determine the cost early-warning index: according to the characteristics of the construction project and the type of “Responsibility Letter for Construction Project Management Objectives,” the feasible target cost is determined, which provides the basis for the process of early warning.
3. Establish the cost early-warning system: including inputting the original data information of completed projects such as target cost, actual cost, cost of each progress node, and construction progress to form a database and inputting the existing projects under construction into the system according to the construction progress so as to facilitate tracking the cost progress of new projects. In addition, exchange and learn from the more advanced cost management measures of similar enterprises and enrich the cases in the database for reference in future work.
4. Monitor and evaluate the process: from the comparison and bidding of suppliers in the construction preparation stage to the monitoring of the authenticity and rationality of cost produced in the construction stage, the analysis of cost change, the identification of early warning, and the risk assessment of settlement in the final stage, the whole process of cost management can be dynamically monitored and evaluated.
5. Organize the cost analysis meeting: hold a cost analysis meeting for the projects that have shut down, and if necessary, adopt the field investigation method to control the latest progress of the project, eliminate abnormal factors, and timely report the projects that are really abnormal to the department leaders.

#### 4.1.2. Organizational Reconstruction

In order to keep the organizational structure of a company's management layer separated from the construction layer unchanged, a cost management center is set up, and the project department submits the cost information of construction to the cost management center for review and then submits it to the corresponding departments for retention and recording. Company A's organizational reconstruction is shown in Figure 3:

### 4.2. Operation Design of Cost Early-Warning System

#### 4.2.1. Systematic Operation Platform

The operation of Company A's cost early-warning system depends on the support and connection of each platform, and its framework should at least include prearrangement, current situation evaluation, trend prediction, and regulation scheme design.

*(1) Prearrangement*. the operating platform of the system should take cost accounting as the starting point, refer to the cost of each subitem listed in the “Construction Project Cost Analysis and Cost Control Table” for accounting. The cost analysis meeting suggests to be organized in time by the cost management center when the construction project is abnormal. The project leader, project management department, and finance department should be invited to participate together, and the cost and output income of the current month need to be compared with the statements and budgets of the previous period, respectively. After the longitudinal analysis, the cumulative amount of the whole project should be analyzed by focusing on the projects with large profits or losses in the process. In addition, the advanced cost management system can provide more accurate and timely feedback on abnormal situations and transmit them to the relevant responsible persons, thus reducing the information transmission time in the middle and effectively improving the work efficiency.

*(2) Evaluation of current situation*. cost early-warning system should work out a reasonable floating range based on the budgeted cost, which can comprehensively consider the cost preference of the project management department. It should also consider the sustainable profitability, capital turnover efficiency, and tax planning of the enterprise in combination with the management status and strategic objectives of the whole company so as to effectively guarantee the operational safety of the enterprise. In addition, outside the reasonable floating range, it is necessary to set the corresponding sensitive range according to different degrees, which can trigger the corresponding early-warning signal in time and facilitate the relevant responsible person to handle it in time.

*(3) Trend prediction*. Company A should establish a systematic mechanism of early-warning display, prediction, and warning at the same time so as to analyze and predict the development trend of future cost through different sensitive intervals of current situation assessment. In addition, the trend should be quickly transmitted to relevant responsible persons to provide data support and guidance for their next construction plan as well as to pay attention to the feedback information and the solutions in time. Moreover, a database of coping strategies corresponding to warning needs to be established to enrich the contents of the database while warning, which can provide reference for the cost management and can be extended to other enterprises in the industry.

*(4) Regulation scheme design*. in the research of cost early-warning system, Company A needs to comprehensively consider factors such as safety production risks and engineering quality risks faced by construction enterprises. The cost problems caused by the complexity and variability of the external environment cannot be solved naturally during the construction process. It is necessary to deeply explore the root causes of cost deviation and find solutions. At the same time, when the enterprises are regulating and controlling the system to solve the existing cost problems, new risks and problems may arise. Therefore, Company A should combine existing and contingent environmental planning measures to solve various difficulties and fully consider the possible adverse effects of existing measures to select the appropriate scheme.

#### 4.2.2. System Operation Program

Company A's operation program of cost early-warning system is divided into four parts: early-warning preparation, cost monitoring and signaling, problem handling, and summary, which is a cycle of continuous self-improvement [29]:

1. Early-warning preparation, that is to determine the possible arrival time of the crisis: including early-warning knowledge reserve, early-warning elements identification and collection, and early-warning index system establishment. First, the establishment of early-warning index system needs to input the existing data of completed projects and calculate the total construction cost and its ratio. It is necessary to distinguish the project department, the nature of the project, and the letters of responsibility so as to determine the early-warning index system of Company A; secondly, enter the “Construction Project Cost Analysis and Cost Control Table” of each project; and finally, the construction in progress is entered into the system together with the contract amount and the existing cost.
2. Cost monitoring and signaling: when the reasonable floating range determined by the project is exceeded, the system will send out a general warning prompt, which will be passed to every member of the cost management center for attention and sent to the project leader. Cost monitoring is divided into two parts: cost operation status monitoring and cost deviation analysis rainbow early-warning chart. Two modes of real-time monitoring and timing monitoring are adopted for monitoring. Real-time monitoring is carried out at every operation with cost. After this operation is completed, the computer software will automatically draw a rainbow early-warning chart, which is convenient for operators to judge. While the timing monitoring is similar to the original mode of Company A, after the quarterly financial statements are prepared, it can be seen that Company A monitors the cost operation status mainly by real-time monitoring, supplemented by regular monitoring. When the rainbow warning chart shows that it exceeds the corresponding precontrol line, it will trigger the warning system and release the corresponding warning signal to the relevant responsible person.
3. Problem handling: when the cost early-warning system sends an early-warning signal, the cost management center starts to analyze the cause. At this time, the person in charge of the project needs to write written materials and report them to the cost management center for explanation. If users go beyond the warning line to the area for shutdown and rectification, it will automatically trigger a severe warning. In principle, no new cost should be added, and the project leader should be immediately notified to hold a cost analysis meeting and discuss the causes and countermeasures together. Any subsequent cost can only be added with the account number of the person, and the cost can only be added normally after the early warning is lifted. After investigating the reasons, it will search the matching solution from the system and implement the action plan to remove the warning signal. When the cause of the problem is not in the system reserve plan, it will seek solutions from outside actively, including communication with owners, government agencies, and suppliers, as well as investigation and reference from other construction enterprises.
4. Summary: after the early warning is lifted, the early-warning treatment plan will be recorded, summarized, and entered. The summary of early warning is generally divided into three types. First, analysis of the cause, which is meant to describe the causes of this crisis. Second, conclusion, where Company A can start from the operation such as early-warning identification and crisis handling or evaluate from the macrostructure such as the layout structure of the whole early-warning system and the establishment of early-warning indicators; finally, rectification. After comprehensively classifying the problems, timely put forward rectification opinions and implement them.

The flow chart of the cost early-warning system is shown in Figure 4.

### 4.3. Establishment of Cost Early-Warning Model

#### 4.3.1. Selection of Indicators

The premise of combining cost management with schedule monitoring is the need for an accurate schedule plan. The work content of the project and the sequence constitute the key factors of the schedule. According to the requirements of the construction budget and scheme, the decomposition structure diagram of the construction operation needs to be constructed. In addition, it should decompose the construction into different task structures and then into different task units according to their interrelation and logical order. Task units need to be integrated into daily production and operation activities to guide the construction projects to be completed according to the schedule.  Figure 5 is a typical diagram of work breakdown structure.

According to the chart, it is more appropriate to bring earned value indicators into the cost early-warning system of Company A after defining the work content and scope of the construction project.

#### 4.3.2. Cordon Setting

There are two kinds of deviations in the process of construction progress, namely, positive deviation and negative deviation. The positive deviation indicates the cost saving or the advance of progress. However, it may also be the result of the decline of engineering quality, or the change of operation plan, which seems to be uncertain and will bring hidden dangers to the next construction progress. Negative deviation often brings the waste of cost or backward progress, but unexpected situations also happen from time to time. For the convenience of later construction, the overbudget expenditure that often happens in the early stage needs specific analysis. Therefore, it needs to comprehensively consider various factors in the construction process.

The cost early-warning system based on deviation analysis is suitable for dynamic monitoring of construction project cost management where the results presented by this system can provide timely and accurate cost dynamic information to relevant responsible persons and provide data support for the follow-up progress of construction projects.

The deviations between the actual schedule and the planned schedule and between the actual cost consumption and the budget consumption cannot cover the complicated actual situation. If the deviation value is extremely small, the correction cost will be high; if the deviation value is large, then active measures should be taken. In addition, other deviations have no corresponding correction; therefore, it is necessary to delimit the range of deviation and establish early-warning system for deviation analysis.

Rainbow early-warning system can realize the above functions. The application of the rainbow early-warning system needs to first determine the deviation unit and early-warning level, then bring different project data into the system for measurement and judgment, and visually display the results, which is convenient for the responsible person to control and take action in time.

Studies have shown that there is no clear specification for the demarcation of the cost warning line. Coupled with the particularity of large size and tight construction period, there is not enough theoretical support in this field [30, 31]. The research on financial early warning follows the principle of “half-and-half division” and delimits the interval according to the cost management requirements of Company A. As shown in Figure 6, with the target value as the control center line, a control line is divided on both sides of the target value, then 0.50 standard deviation is taken as the unit to form a control area of standard value, which is called the target area (blank area). Afterwards, take the target value as the control center line, draw a warning line on each side of the blank area, and form an area with a difference of 0.5 standard deviation from the boundary line of the target area, which is called the warning area (light grey area). When reaching the alert zone, a general warning signal requires the cost management center to contact the project department in time so as to understand the progress of the project and avoid the potential risks in the construction process. In addition, a cost analysis meeting will be organized if necessary. Outside the two light grey areas, it is the shutdown and rectification area (dark grey area). When reaching the shutdown and rectification zone, it is considered that the current scheme cannot meet the actual needs. If the cost is out of control, a severe shutdown warning signal will be sent immediately, and the cost management center should organize a cost analysis meeting to eliminate the problems before resuming the construction of the project.

#### 4.3.3. Cost Warning Boundary

Because the deviation of cost does not involve whether the work is in the critical path, the monitoring of cost early warning is better than that of progress early warning. The dynamic early warning of engineering construction project cost can be adjusted according to the tracked deviation to determine whether measures need to be taken and whether the cost plan needs to be adjusted.

Set the deviation strength value of the cost as follows:

(1) $$\begin{array}{c} ai=\frac{\text{BCWP}*\text{ACWP}}{\text{ACWP}}\times 10\times \frac{\text{CV}}{\text{ACWP}}\times 100\%\text{.} \end{array}$$

Assuming that the control range of allowable fluctuation of the project cost is ±*δ*±*δ*; , the boundary for monitoring and warning signals is ±*ε*, which is divided into the following four situations for analysis.

1. If the cost deviation intensity *αi* falls beyond +*δ*, the cost plan needs to be revised
2. If the cost deviation intensity *αi* falls beyond −*δ*, it is necessary to consider whether the cost balance has an impact on the project quality based on the project situation
3. If the cost deviation intensity *αi* falls between +*δ* and +*ε*, an early warning is needed to find out the key factors leading to the deviation and take measures to reduce the cost
4. In other cases, it is considered that the cost is within the controllable range, so no treatment is required.

## 5. Conclusion

For enterprises, choosing the best cost management system according to their actual situation and the degree of management refinement can promote the management level of enterprises. This paper attempts to set up a cost early-warning system for construction projects by setting up a cost control center. The results show that the earned value management method is helpful to establish the key points of cost early warning, set the warning line index, and establish the cost warning boundary so as to meet the actual situation of the company and construct an effective construction project cost early-warning system. The cost early-warning system can realize the dynamic control of the whole process of the cost before, during, and after the project, where the cost status more intuitively and in the whole process is displayed and warned, which is convenient to compare and analyze different construction projects.

## Figures and Tables

**Figure 1:** Implementation stage of the construction project.

**Figure 2:** Main parameters in EVM.

**Figure 3:** Organizational reconstruction of Company A.

**Figure 4:** Design of cost early-warning system.

**Figure 5:** Work breakdown structure diagram.

**Figure 6:** Rainbow diagram.

**Table 1:** Evaluation index of earned value management.

Index	Calculation formula	Judging procedure
CV	CV = BCWP − ACWP	Measure the level of cost management. If CV < 0, it means that the project operation cost exceeds the expenditure; If CV ≥ 0, it means that the project operation cost saves expenses.

SV	SV = BCWP − BCWS	Measure the progress of the project. If SV < 0, it means that the project progress is delayed; If SV ≥ 0, it means that the project progress is ahead of schedule.

CPI	CPI = BCWP/ACWP	Measures the execution level of the project budget. If CPI < 1, it means that the cost exceeds the expenditure; If CPI ≥ 1, it means cost savings.

SPI	SPI = BCWP/BCWS	Measure the actual execution level of the project workload. If SPI < 1, the actual progress is insufficient; If SPI ≥ 1, it means that the actual progress is ahead.

## Data Availability

The data set can be accessed upon request.
